# PEGylated Doxorubicin Prodrug-Forming Reduction-Sensitive Micelles With High Drug Loading and Improved Anticancer Therapy

**DOI:** 10.3389/fbioe.2021.781982

**Published:** 2021-11-19

**Authors:** Dongdong Wang, Xiaoyi Zhang, Bingbing Xu

**Affiliations:** ^1^ Minimally Invasive Interventional Therapy Center, Qingdao Municipal Hospital Affiliated to Qingdao University, Qingdao, China; ^2^ Department of Oncology, Qingdao Municipal Hospital Affiliated to Qingdao University, Qingdao, China; ^3^ School of Pharmacy, Shihezi University, Shihezi, China; ^4^ Sports Medicine Department, Beijing Key Laboratory of Sports Injuries, Peking University Third Hospital, Beijing, China; ^5^ Institute of Sports Medicine of Peking University, Beijing, China

**Keywords:** reduction-sensitive, micelles, disulfide, biocompatible, drug delivery

## Abstract

Significant efforts on the design and development of advanced drug delivery systems for targeted cancer chemotherapy continue to be a major challenge. Here, we reported a kind of reduction-responsive PEGylated doxorubicin (DOX) prodrug via the simple esterification and amidation reactions, which self-assembled into the biodegradable micelles in solutions. Since there was an obvious difference in the reduction potentials between the oxidizing extracellular milieu and the reducing intracellular fluids, these PEG–disulfide–DOX micelles were localized intracellularly and degraded rapidly by the stimulus to release the drugs once reaching the targeted tumors, which obviously enhanced the therapeutic efficacy with low side effects. Moreover, these reduction-sensitive micelles could also physically encapsulate the free DOX drug into the polymeric cargo, exhibiting a two-phase programmed drug release behavior. Consequently, it showed a potential to develop an intelligent and multifunctional chemotherapeutic payload transporter for the effective tumor therapy.

## Introduction

Biodegradable nanoparticles with low side effects are intensively employed as potential candidates for the targeted tumor chemotherapy because they can promote the drug solubility in solutions, prolong the circulation time with high stability, enhance the pharmacokinetic property, keep the bioavailability, and improve the tumor accumulation and therapeutic effects by the enhanced permeability and retention (EPR) effect (Lyass et al., 2000; Lukyanov and Torchilin, 2004; Torchilin, 2006; Chao et al., 2012; Huang et al., 2018; Sun et al., 2019). However, low drug loading capacity and incomplete drug release greatly limited the tumor therapy because of the unpredictable drug release by physical encapsulation from the nanoparticles to the cytoplasm. Therefore, stability, drug loading, and stimuli-triggered drug release should be considered for the fabrication of intelligent carriers to improve the tumor chemotherapy.

Doxorubicin (DOX) is an FDA-approved and a typical anticancer drug for the tumor treatment, but it possesses obvious disadvantages in truly clinical application, such as severe toxicity, low bioavailability, and high dose requirement. Therefore, the development of DOX-based drug delivery system has been focused by many studies to simultaneously require the high drug utilization and low side effects (Li et al., 2016; Bao et al., 2019; Fan et al., 2019; Wang et al., 2019; Cytryniak et al., 2020; Zhu et al., 2021). Among the various drug carriers, physical encapsulation and chemical conjugates are two main strategies for the fabrication of drug delivery. Although DOX-loaded carriers have been applied for many applications, they possess many inherent shortcomings like low drug loading, premature burst release, and insensitive manipulation, which are mainly attributed to the high hydrophilicity of DOX drugs. In contrast, polymer conjugates have made great progress on account of their simple architectural design, feasible preparation method, and smart functional fabrication, which provides an alternative for the cancer chemotherapy (Hu and Jing, 2009; Chytil et al., 2012; Hu et al., 2012; Li et al., 2020; Song et al., 2021).

Driven by an urgent requirement to rapid release payloads in response to an intrinsic biological signal, stimulus-sensitive systems have been explored and investigated extensively in the recent years (Wang et al., 2016; Wang et al., 2017; Wang et al., 2018; Zhang et al., 2020a). Among the various stimuli-sensitive carriers, reduction-sensitive micelles have received great attention for intracellular drug delivery on the account of the obvious concentration distinction in the redox potential between the oxidizing extracellular milieu and the reducing intracellular fluids. Reducing glutathione (GSH) is the most abundant reducing molecule with the millimolar concentrations in the intracellular compartments and micromolar concentrations in the extracellular environment. In view of a high reducing potential within the tumor cells and tissues, various reduction-sensitive polymeric nanoparticles have been explored for triggered anticancer drug release. These reduction-responsive nano-systems have demonstrated several unique features, for example, good stability under physiological environment, fast response to intracellular reducing conditions, triggering drug release in the cytosol and cell nucleus, and significantly improved antitumor activity. Accordingly, the disulfide-containing polymeric micelles can maintain stability under physiological conditions in the circulation stage and facilitate intracellular drug release within the tumors by the cleavage of disulfide bonds (Jiang et al., 2011; Sun et al., 2014; Yang et al., 2014; Chen et al., 2015; Cui et al., 2015; Cheng et al., 2017; Cao et al., 2018; Zhang et al., 2019; Zhang et al., 2020b; Li et al., 2020; Zhu et al., 2021).

In this study, we prepared an amphiphilic polymer drug conjugate (PEG–disulfide–DOX) with high and fixed DOX loading content through the mild esterification and amidation reactions (Figure 1), which could self-assemble into the reduction-sensitive micelles in solutions. The bridged disulfide linkages endowed the PEGylated micelles with structural integrity at normal physiological condition but quickly disassemble in response to reductive environment. CCK-8 assays verified the favorable antitumor activity of these PEG–disulfide–DOX micelles. Importantly, in addition to the chemical linkage of DOX drugs, these PEGylated micelles could also encapsulate the free DOX drug into the nanoparticles to further improve the drug loading capacity, exhibiting a programmed DOX release behavior with a long treatment period and an enhanced therapeutic effect.

**FIGURE 1:** Synthetic scheme of the PEG–disulfide–DOX polymer and micelles with reduction-sensitive behavior for intracellular drug release.

## Materials and Methods

### Materials

Poly(ethylene glycol) methyl ether (PEG-OH, M_n_ = 750 g/mol, Alfa Aesor), 3,3′-dithiodipropionic acid (98%, Energy Chemical), 1-(3-dimethylaminopropyl)-3-ethylcarbodiimide hydrochloride (EDCI, 99%, Energy Chemical), 4-(dimethyl-amino)-pyridine (DMAP, 99%, Aldrich), 1,4-dithiothreitol (DTT, 99%, Energy Chemical), triethylamine (TEA, 99%, Beijing Chemical Works), hydrochloric acid, anhydrous magnesium sulfate, and ether were purchased from Beijing Chemical Works. Doxorubicin·HCl (DOX·HCl) was purchased from Beijing Huafeng United Technology Corporation and used as received. Tetrahydrofuran and dimethylformamide were purified by stirring over calcium hydride for 48 h. The cells were supplied by China Infrastructure of Cell Line Resource.

### Characterizations

Nuclear magnetic resonance (NMR) spectra were recorded on a Bruker 400-MHz spectrometer with deuterated chloroform (CDCl_3_) as the solvent. The transmission electron microscopy (TEM) images were obtained on a JEM-2200FS microscope (JEOL, Japan). Dynamic light scattering (DLS) measurements were performed in an aqueous solution using a Malvern Zetasizer Nano S apparatus equipped with a 4.0 mW laser operating at *λ* = 633 nm. All samples of 1 mg/ml were measured at 20°C and at a scattering angle of 173°C. All data were averaged over three times. The fluorescence measurement was carried on a Hitachi F4600 photo-luminescent spectrometer with a xenon lamp as a light source. The confocal laser scanning microscopy (CLSM) images were obtained on a Zeiss LSM 510 microscope.

### Synthesis of the PEG–disulfide–COOH Polymer

PEG-OH (0.75 g, 1 mmol), EDCI (1.2 g, 6 mmol), 3,3′-dithiodipropionic acid (1.22 g, 6 mmol), and DMAP (125 mg, 1 mmol) were dissolved in 50 ml of freshly dried THF solution under a nitrogen atmosphere. After continuous stirring for 24 h at room temperature, the crude products were resolved in DCM and washed with 2 M HCl aqueous solution, saturated NaCl aqueous solution, and DI water for three times and dried over anhydrous MgSO_4_. The final product was precipitated into cool ether for several times to afford the white PEG–disulfide–COOH with 78.1% yields.

### Synthesis of the PEG–disulfide–DOX Polymer

PEG–disulfide–COOH (0.19 g, 0.2 mmol), DOX·HCl (0.3 g, 0.5 mmol), and TEA (70 μl, 0.5 mmol) were dissolved in 20 ml of freshly dried DMF under a nitrogen atmosphere. After continuous stirring for 24 h at room temperature, the crude products were resolved in DCM and washed with 2 M HCl aqueous solution, saturated NaCl aqueous solution, and DI water for several three times and dried over anhydrous MgSO_4_. The final product was precipitated into ether for several times to afford the dark-red PEG–disulfide–DOX with 58.4% yield.

### Formation and Self-Assembly of the Polymeric PEG–disulfide–DOX Micelles and DOX-Loaded PEG–disulfide–DOX Nanoparticles

5 mg of PEG–disulfide–DOX was dissolved in 1 ml of DMF, and then 4 ml of deionized water was added dropwise into the solution at the rate of 0.05 ml/min via a syringe pump. The colloidal dispersion was further stirred for another 4 h at room temperature. Afterward, the organic solvent was removed by dialysis (MW cutoff, 1 kDa) against deionized water for 3 days. These PEG–disulfide–DOX micelles were obtained and recorded by the TEM and DLS measurements.

5 mg of PEG–disulfide–DOX was dissolved in 1 ml of DMF, followed by adding a predetermined amount of free DOX·HCl and 2 molar equivalents of triethylamine. Then, 4 ml of deionized water was added dropwise into the solution at the rate of 0.05 ml/min via a syringe pump. The colloidal dispersion was further stirred for another 4 h at room temperature. Afterward, the organic solvent and free DOX was removed by dialysis (MW cutoff, 1 kDa) against deionized water for 3 days. These DOX-loaded PEG–disulfide–DOX nanoparticles were obtained and recorded by the TEM and DLS measurements.

### Stability and Reduction-Sensitive Destabilization

For determining the reduction-sensitive destabilization of PEG–disulfide–DOX micelles and DOX-loaded PEG–disulfide–DOX nanoparticles, a certain amount of phosphate buffered saline (PBS) with and without DTT (10 mM) was, respectively, added into the abovementioned polymeric nanoparticles (1 mg/ml) at 37°C in a shaking water bath. After treatment for various times, morphological and dimensional changes were recorded by TEM and DLS measurements.

### *In vitro* Drug Release

Reduction-triggered DOX release measurement was conducted as below: dispersed PEG–disulfide–DOX micelles and DOX-loaded PEG–disulfide–DOX nanoparticles were, respectively, added into a dialysis membrane tube (MW cutoff, 1 kDa), which was then incubated in PBS with and without DTT (10 mM) solutions at 37°C in a shaking water bath. The reduction-triggered DOX-released profiles were determined by measuring the UV-vis absorbance of solutions at 480 nm. The release experiments were conducted in triplicate and the results were expressed as average data with standard deviations.

### Cell Culture, Cellular Uptake, and Intracellular Localization

MCF-7 cells were plated on microscope slides in a 96-well plate (1 × 10^4^ cells/well) using DMEM (Dulbecco’s Modified Eagle Medium) containing 10% FBS (fetal bovine serum) and antibiotics (50 units/mL penicillin and 50 units/mL streptomycin) at 37°C in a humidified atmosphere containing 5% CO_2_. After incubation for 24 h, the predetermined amounts of free DOX and PEG–disulfide–DOX nanoparticles (equivalent to free DOX) were added for 2 h at 37°C. After removal of the culture medium, the cells were washed for three times with PBS. Finally, after fixing with 4% paraformaldehyde, the MCF-7 cells were observed by a CLSM with excitation at 488 nm for DOX.

### Activity Analyses

Cytotoxicity of polymeric PEG–disulfide–DOX micelles and DOX-encapsulated PEG–disulfide–DOX nanoparticles was studied *in vitro* by the CCK-8 assay. The MCF-7 cells were seeded onto a 96-well plate at a density of 1 × 10^4^ cells per well in 200 μl of medium containing 10% FBS and incubated for 24 h. The medium was replaced by 90 μl of fresh DMEM medium containing 10% FBS, followed by adding various concentrations of micelle suspensions. After incubation for another 24 h, the culture medium was removed from the cell culture plates, and 100 μl of fresh culture medium and 10 μl of CCK-8 kit solutions were immediately mixed for another 4 h of incubation. Finally, 100 μl of solutions were put into a 96-well plate. The optical density of each well at 450 nm was read by a microplate reader. The cells cultured in the DMEM medium containing 10% FBS (without exposure to micelles) were used as controls. The data were expressed as average ± standard deviations (*n* = 5).

## Results and Discussion

### Synthesis of PEG–disulfide–DOX Prodrugs

The reaction scheme for the synthesis of the disulfide-bonded PEGylate DOX prodrug was illustrated in Figure 1. Based on the simple esterification reaction of 3,3′-dithiodipropionic acid and sequential amidation reaction of DOX, the PEG–disulfide–DOX was feasibly synthesized by the ^1^H NMR spectra. Figure 2A clearly exhibited the typical resonance signal assignments of PEG–SS–COOH polymer, and the integration ratio of typical resonance peaks (I_a_/I_c_/I_d_) was extremely close to 3:2:4, confirming the intact structure of well-defined PEG–disulfide–DOX polymer. On account of the complicate peaks of the DOX drug, it was not provided with a clear representative peak assignment. After the chemical linkage of DOX via the amidation reaction, the integrated assignments of PEG (*δ* 3.3 ppm and 3.5–4.1 ppm) and DOX moieties (red signals) were observed as in Figure 2B. Especially, the shift of the typical characteristic peaks of *d,e* indicated the chemical conjugation of PEG chain and DOX drug with the identical structure.

**FIGURE 2:** ^1^H NMR spectra of **(A)** PEG–SS–COOH and **(B)** PEG–disulfide–DOX polymers. The shift peaks and the intricate peaks of DOX components verify the polymeric preparation.

### Preparation, Stability, and Reduction-Sensitive Destabilization of PEG–disulfide–DOX Micelle

In aqueous solutions, the amphiphilic PEG–disulfide–DOX polymers could self-assemble into micelles. The TEM image in Figure 3A-a showed spherical structures with a size of ca. 78 nm, while the DLS result in Figure 3B-a displayed the z-average particle size of ca. 162 nm and a polydispersity index of 0.18. The size difference was attributed to the swelling state of PEG–disulfide–DOX in solutions compared to the dry state by TEM. Since the diameter was less than 200 nm, the PEG–disulfide–DOX micelles were suitable to maintain the lowered RES uptake level and minimal renal excretion, indicating their potential application as a smart drug carrier to enhance the passive tumor-targeting capacity by the EPR effect. On account of the stable disulfide linkages between the hydrophobic DOX and the hydrophilic PEG in mild conditions, the PEG–disulfide–DOX micelles maintained the satisfactory storage stability for the drug formulations. To ensure the high-effective intracellular drug release, it is important for stimuli-responsive prodrugs to meet the requirements of precise target ability and controllable drug release within the target cells upon changes in physical and chemical environments. The reduction-sensitive disulfide linkers can make the PEG–disulfide–DOX micelles susceptible to disassemble in the presence of 10 mM DTT solutions. After incubation of 2 h in 10 mM DTT solutions, the uniform structures gradually degraded into small aggregates, as in Figure 3A-b. In addition, Figure 3B-b exhibited the size variation with the occurrence of the small size of molecules and large size of aggregates, confirming the redox-induced cleavage of disulfide bonds and dissociation of the polymeric micelles. Moreover, the diameter variations of PEG–disulfide–DOX micelles in PBS solutions were characterized using DLS, revealing their better storage stability over 48 h in Figure 3C. Once when incubated in the reductive DTT solutions, these PEG–disulfide–DOX micelles were quickly degraded with the gradual occurrence of small PEG chains and large hydrophobic DOX drugs over time as observed in Figure 3D, which indicated that these kinds of reduction-sensitive micelles could maintain colloidal stability under extracellular conditions and were prone to rapid dissociation under redox-stimuli mimicking the intracellular conditions.

**FIGURE 3:** **(A)** TEM images and **(B)** size changes of the PEG–disulfide–DOX micelles before (a) and after (b) treatment of 10 mM reducing agent of DTT solutions for 4 h. **(C)** Size variations of the PEG–disulfide–DOX micelles after treatment in PBS (pH = 7.4) solutions. **(D)** Size variations of the PEG–disulfide–DOX micelles after treatment of 10 mM reducing agent of DTT solutions for various times. The PEG–disulfide–DOX micelles possessed reduction-responsive degradation in a high concentration of reductive agents, but displayed good stability at physiological conditions for a long period.

### Loading and *in vitro* Drug Release of DOX

Based on the chemical linkage of DOX, the drug loading content in the PEG–disulfide–DOX prodrug was precisely calculated to be 37.1 wt%, which was higher than most of the other reported DOX prodrugs for therapeutic usage. The drug release profile of PEG–disulfide–DOX micelles was performed under the physiological conditions (PBS, pH 7.4) and the reductive DTT agents (PBS, pH 7.4, 10 mM) to simulate in the intracellular environment with a high reduction in the cytoplasm and the cell nucleus at 37°C. In contrast to a negligible DOX release in pH 7.4 solutions, PEG–disulfide–DOX micelles could quickly release the DOX drugs in 10 mM of reducing DTT agents, exhibiting a high release content of 86.9% at 24 h (Figure 4). This phenomenon was attributed to the cleavage of disulfide bonds and acceleration of the DOX release. Such variations suggested that the PEG–disulfide–DOX micelles could maintain stability and eliminate the premature burst release in blood circulation, thus effectively promoting the DOX release from polymeric prodrugs during the process of intracellular trafficking. In contrast to the conventional liposomal DOX formulations with poor stability and premature drug burst release, these reduction-sensitive micelles with feasible preparation, good water stability, passive tumor-targeting ability, and controlled drug release would be developed as clinical products with advanced tumor endocytosis and enhanced therapeutic effect.

**FIGURE 4:** Reducing agent of DTT-triggered DOX release from PEG–disulfide–DOX micelles with or without DTT (10 mM) solutions at 37°C. The drug release profile reflects the reduction response of the micelles with good stability in neutral environment and quick dissociation in reductive agents.

### Cellular Uptake, Intracellular Localization, and *in vitro* Antitumor Activity

Polymeric micelles can escape from endosomes and transport into cytoplasmic organelles. In order to assess the internalization of PEG–disulfide–DOX prodrugs, cellular uptake and intracellular drug release were first estimated by MCF-7 cells using CLSM. As shown in Figure 5, the appearance of the red DOX fluorescence was observed at the cytoplasm within the cells after incubation for 2 h, indicating that the PEG–disulfide–DOX nanoparticles were easily internalized within the cells and concentrated in the nuclei via the endocytosis process. These findings also indicated that the efficient DOX release from the nanoparticles into the nucleus, revealing the applicability and practicability of drug delivery. Furthermore, we estimated the *in vitro* antitumor activity of PEG–disulfide–DOX micelles using MCF-7 cells. The CCK-8 assay exhibited that after incubation for 24 h, these micelles could effectively inhibit the cell growth with high antitumor activity toward MCF-7 cells. In addition, it was found that the PEG–disulfide–DOX micelles exhibited similar antitumor activity compared to the free DOX in the low concentration but displayed lower toxicity in high concentration. This may describe the feasible permeation of small DOX molecules into the cellular and nuclear membranes via the passive diffusion effect, while the PEG–disulfide–DOX micelles were first prone to be endocytosed to the cells and then dissociated to release the DOX drugs in the cytosol and nucleus. So, these internalization processes slowed the pace for inhibiting the tumors, by which PEG–disulfide–DOX micelles can express the precise target ability and controllable drug release inside the targeted tumors.

**FIGURE 5:** **(A)** CLSM of MCF-7 cells after incubation with PEG–disulfide–DOX micelles for 2 h; a: bright field image, b: red fluorescence image, and c: overlap of bright field and fluorescence images. **(B)** Cytotoxicity of MCF-7 cells following 24-h incubation with PEG–disulfide–DOX and free drugs as a function of DOX dosages. The data are presented as the average ± standard deviation (*n* = 5).

### Fabrication of DOX-Encapsulated PEG–disulfide–DOX Nanoparticles

To actually simulate the tumor environment and achieve the maximum tumor inhibition, it is necessary to maintain effective drug concentration and prolong drug activity at various periods for improving the therapeutic effects. Therefore, chemically linked prodrugs were not intelligently activated to rapidly kill the tumors at the early stage, which required the design and fabrication of a smart criterion that can meet the high drug concentration to kill the tumors at an early period and exert stimuli-responsive effects upon changes in the target cells for a long period. Consequently, it is necessary to further encapsulate the free DOX drug into the PEG–disulfide–DOX micelles to generate a drug delivery system with the synergistically physical encapsulation and chemical conjugation interactions, which showed the rapid release of encapsulated drugs to enhance the local drug concentration within a short time, followed by the release of conjugated drugs to continue the effective treatment over a longer period, thereby resulting in improved therapeutic effect. In this case, the DOX-loaded PEG–disulfide–DOX could not only discharge the interior DOX to maintain the intracellular DOX concentration at the initial phase but also release the conjugated drug to effectively kill the tumors to promote the therapeutic effect, thus achieving a programmed drug release behavior with high-efficient antitumor activity.

By means of the solution’s self-assembly strategy, free DOX molecules were feasibly loaded in the micelles to form the DOX-loaded PEG–disulfide–DOX nanoparticles. As shown in Figures 6A,B, the self-assembles could still maintain the spherical morphologies with the increscent diameters. Moreover, Figure 6C showed that the DOX-loaded PEG–disulfide–DOX nanoparticles exhibited a two-phase programmed drug release behavior compared to that of PEG–disulfide–DOX micelles in Figure 4, which testified that the physically loaded DOX could release at an early period to achieve high drug concentration to kill the tumors, and the conjugated DOX provided a responsive drug release to prolong the treatment period. Compared to the free DOX and PEG–disulfide–DOX nanoparticles, these DOX-encapsulated PEG–disulfide–DOX nanoparticles possessed more advanced capacities with high drug loading, sufficient drug release, and enhanced therapeutic effects of antitumor activity toward MCF-7 cells after the incubation of 24 h (Figure 6D). It was mentioned that the physical drug loading content did not need too much high concentration because of the undesirable drug release that may cause potential side effects. Besides, other hydrophobic drugs could be also encapsulated into these nanoparticles to acquire the novel drug combination, which may be more promising to enhance therapeutic effects and satisfy the clinical requirements.

**FIGURE 6:** **(A)** TEM image, **(B)** DLS result, and **(C)** *in vitro* drug release profile of DOX-encapsulated PEG–disulfide–DOX nanoparticles with or without 10 mM DTT solutions. **(D)** Cytotoxicity of MCF-7 cells following 24-h incubation with DOX-encapsulated PEG–disulfide–DOX aggregates as a function of DOX dosages. All the data are presented as the average ± standard deviation (*n* = 5). These DOX-encapsulated PEG–disulfide–DOX nanoparticles possessed capacities with high drug loading, sufficient drug release, and enhanced therapeutic effects of antitumor activity.

## Conclusion

In summary, we developed a PEGylated doxorubicin prodrug via the conjugated hydrophobic DOX into a short PEG chain through the cleavable disulfide linkages. These PEG–disulfide–DOX micelles could maintain the structural integrity and stability, reserve high drug loading content, and tailor the drug release. The liable disulfide links endowed the PEG–disulfide–DOX prodrugs with a reduction-sensitive ability to achieve the controllable drug release inside the target cells. After treatment with reducing DTT agents, the uniform PEG–disulfide–DOX micelles could quickly dissociate into the microsized particles and severe aggregations to release the DOX drugs. *In vitro* cytotoxicity results demonstrated these PEG–disulfide–DOX micelles possessed a fast internalization and drug release capacity to effectively inhibit the growth of MCF-7 cells, demonstrating the favorable antitumor activities. In addition, this kind of nanoparticle could further encapsulate small free DOX drugs or other biological molecules, which can be developed as the novel translational DOX formulations and with advanced multifunction in drug delivery systems. Thus, we believe that these prodrug nanomedicines will hold promise to an alternative translational DOX formulation for cancer chemotherapy.

## Data Availability

The raw data supporting the conclusion of this article will be made available by the authors, without undue reservation.
